# Mechanisms of Qing-Gan Li-Shui Formulation in Ameliorating Primary Open Angle Glaucoma: An Analysis Based on Network Pharmacology

**DOI:** 10.1155/2022/8336131

**Published:** 2022-07-20

**Authors:** Lin Mu, Zhiguo Dong, Yinjian Zhang

**Affiliations:** Department of Ophthalmology, Longhua Hospital Shanghai University of Traditional Chinese Medicine, Shanghai 200032, China

## Abstract

**Objective:**

In this study, we investigated the mechanism of Qing-Gan Li-Shui formulation (QGLSF) in treating primary open glaucoma (POAG) by network pharmacology and *in vitro* experiments.

**Methods:**

The active pharmaceutical ingredients (APIs) of GLQSF (prepared with *Prunella* vulgaris, Kudzu root, *Plantago asiatica*, and *Lycium barbarum*) were obtained from the Traditional Chinese Medicine Systems Pharmacology Database and Analysis Platform (TCMSP) and Yet Another Traditional Chinese Medicine database (YATCM). The targets of POAG were screened out with GeneCards, OMIM, PharmGKB, Therapeutic Target Database (TTD), and DrugBank databases. The Venny platform was used to summarize the core targets. Topological analysis was performed using Cytoscape3.8.0. A protein-protein interaction network was plotted by STRING online. The key targets were subjected to GO and KEGG enrichment analyses. Finally, the effects of APIs were verified by a model of chloride hexahydrate (CoCl_2_)-induced retinal ganglion cells-5 (RGC-5).

**Results:**

The main APIs were selected as quercetin (Que) by network pharmacology. Nine clusters of QGLSF targets were obtained by the PPI network analysis, including AKT-1, TP53, and JUN. KEGG enrichment analysis showed that these targets were mainly involved in the AGE-RAGE signaling pathway. By *in vitro* experiments, Que promoted cell proliferation. The secretion of AKT-1, TP53, JUN, AGE, and RAGE in the cell culture supernatant decreased, as shown by ELISA. The mRNA levels of AKT-1, TP53, JUN, and RAGE decreased, as shown by RT-PCR. QGLSF may employ the AGE-RAGE signaling pathway to counter POAG.

**Conclusion:**

This study preliminarily elucidates the efficacy and mechanism of QGLSF in the treatment of POAG.

## 1. Introduction

Primary open glaucoma (POAG) is a leading cause of irreversible blindness worldwide [1]. In its early phase, intraocular pressure rises, resulting in atrophy of optic nerve axons, blockade of axoplasmic flow, insufficient nutrient supply to retinal ganglion cells (RGCs), and even subsequent injury of optic nerve fibers [2]. At present, POAG can be controlled through reducing intraocular pressure [3]. If intraocular pressure control is unsatisfactory, surgical treatments are required, such as laser plasty and resection [4]. Despite these efforts, many patients still experience progressive visual field loss.

Traditional Chinese medicine (TCM) has shown clinical efficacy against POAG [5]. Qing-Gan Li-Shui formulation (QGLSF) is composed of *Prunella* vulgaris, Kudzu root, *Plantago asiatica*, and *Lycium barbarum*. Experimental studies have shown that QGLSF can reduce intraocular pressure and inhibit the apoptosis of retinal ganglion cells (RGCs) in a rat model of microbead-induced chronic intraocular hypertension [6]. Network pharmacology can be adopted to analyze the active pharmaceutical ingredients (APIs) and targets of TCM formulations, thus providing insight into the therapeutic mechanisms of TCM from a systemic perspective [7, 8].

RGC-5 was first regarded as a cell line derived from rat retinal ganglion cells, but recent studies have shown that it corresponds to the mouse photoreceptor cell line 661W [9]. Despite such contamination, studies have shown that RGC-5 can still be used to test hypotheses about neural cells derived from retinal cell lines [10–12]. An *in vitro* model of chloride hexahydrate (CoCl_2_)-induced hypoxic damage in retinal ganglion cells-5 (RGC-5) reveals the pathological mechanism of glaucoma [13, 14]. It has been found that CoCl_2_ regulates specific genes to induce hypoxia [15].

In this study, we used the network pharmacology method to explore the potential APIs and targets of QGLSF in the treatment of POAG. The RGC-5 hypoxia injury model was established to validate the functions of key APIs and their targets.

## 2. Materials and Methods

### 2.1. Screening APIs and Targets of QGLSF

Based on the TCMSP database (https://old.tcmsp-e.com/tcmsp.php) and the YATCM database (https://cadd.pharmacy.nankai.edu.cn/yatcm/home), the APIs in QGLSF were searched according to oral bioavailability (OB) ≥30% and drug likeness (DL) ≥0.18. The targets of QGLSF were screened out of the TCMSP. UniProt database (https://www.uniprot.org).

### 2.2. Screening Genes Related to POAD

The key words “primary open angle glaucoma” were searched in GeneCards database (https://www.genecards.org), OMIM database (https://omim.org), PharmGKB database (https://www.pharmgkb.org), TTD database (https://db.idrblab.net/ttd) and Drugbank database (https://go.drugbank.com) databases for the genes related to POAG. All relevant data were downloaded, and duplicates were eliminated.

### 2.3. Predicting the APIs, Targets, and Pathways of QGLSF

The genes targeted by POAG and QGLSF were imported into the VEENY 2.1.0 database (https://bioinfogp.cnb.csic.es/tools/venny/index.html). The PPI network of these genes was constructed by STRING 2.1.0 (https://bioinfogp.cnb.csic.es/tools/venny/index.html). Hub genes were determined by CytoNCA plugin. Topological analysis was performed using Cytoscape3.8.0 to visualize the regulatory network of the APIs. GO and KEGG enrichment analyses were performed by R (version4.0.2).

### 2.4. Drugs and Reagents

Quercetin was purchased from Absin Biosciences Co., Ltd (Shanghai, China); fetal bovine serum and penicillin-streptomycin from Gibco (Carlsbad, USA); Dulbecco's modified eagle's medium (DMEM) high glucose medium and trypsin solution from Cytiva HyClone (USA); dimethyl sulfoxide (DMSO) and cobalt (II) chloride hexahydrate (CoCl_2_) from Sigma Chemicals (St.Louis, USA); Cell Counting Kit-8 from Dojindo (Kumamoto, Japan); FITC Annexin V Apoptosis Detection Kit1 from ThermoFisher Scientific (Waltham, USA); MitoTracker Red CMXRos from Cell Signaling Technology (Danvers, USA); RAT AGEs, RAGE, JUN, AKT1, and TP53 ELISA KIT from Shanghai Lengton Biosciences Co., Ltd (Shanghai, China); DAPI and TriQuick reagent from Beijing Solarbio Scienceamp Technology Co., Ltd. (Beijing, China); TRIzol reagent from Invitrogen (Carlsbad, USA); Prime Script™ RTMasterMix from TaKaRa (DaLian, China); and SYBR Qpcr Master Mix from Vazyme (NanJing, China).

### 2.5. Cell Culture

Rat retinal ganglion cells (RGC-5) were purchased from the American Type Culture Collection (Manassas, USA). The cell culture medium consisted of 10% fetal bovine serum, 1% penicillin-streptomycin, and DMEM. Cells were grown at 37°C in an incubator with 5% CO_2_ and 95% air, and passaged once having grown to 70–80% confluence.

### 2.6. Cell Modeling and Treatment

Quercetin (Que) was completely dissolved in DMSO and diluted with cell culture medium at different concentrations for later use. CoCl_2_ was completely dissolved in DMSO. The CoCl_2_ solution was prepared at a final concentration of 600 *μ*M, based on the dose of CoCl_2_ used in previous studies [16]. As a vehicle, the final level of DMSO in the culture medium was 0.05% (v/v). RGC-5 cells at passages 10–25 were selected and seeded at 2 × 105/ml in six-well plates for 24 h. Afterwards, the medium containing Que (25 *μ*M) was added and incubated for 24 h, followed by an incubation for 24 h containing CoCl_2_ to induce hypoxic injury.

### 2.7. Cell Viability Assay

The cells were seeded in 96-well plates (1 × 104/ml) for 24 h. After drug intervention, 10 *μ*l of CCK-8 solution was added to each well and incubated for 1 h at 37°C in the dark. Absorbance was measured at 450 nm using a microplate reader.

### 2.8. Apoptosis Assay

After cell modeling, the cells were washed with PBS and resuspended in 200 *μ*l of binding buffer. Then, 5 *μ*l of Annexin V–FITC was added and incubated for 10 min at room temperature. After the cells were washed with binding buffer and resuspended, 10 *μ*l of propidium iodide staining solution was added for 5 min. Flow cytometry was used to detect the apoptosis of cells.

### 2.9. Cell Supernatant

After cell modeling, the cell culture supernatant was collected and centrifuged at 3000 rpm/min for 20 min. Next, 50 *μ*l of cell culture supernatant and 50 *μ*l of biotin antigen were added to each enzyme-labeled coated well and incubated at 37°C for 30 min. After washing for five times with washing solution, 50 *μ*l of avidin-HRP was added to each well, incubated at 37°C for 30 min, and washed for another five times. The developer solution was added to each well and incubated at 37°C in the dark for 10 min before the addition of the stop solution. The absorbance was detected by a microplate reader at a wavelength of 450 nm.

### 2.10. mRNA Detection

The TRIzol method was used to extract RNA from samples. RNA was reverse-transcribed into cDNA with PrimeScript RT, followed by PCR amplification with gene-specific primers. Primer sequences and product lengths are shown in Table 1. The GAPDH was used as a control for unification and the results were calculated using the 2^‒ΔΔCt^ method.

### 2.11. Statistical Analysis

Statistical analysis was performed using GraphPad8. Multiple-group comparison was performed through one-way analysis of variance. A between-group comparison was performed through *t*-tests. All experimental data were expressed as mean ± SD. Statistical significance was considered when *p* < 0.05.

## 3. Results

### 3.1. APIs and Targets of QGLSF

QGLSF was mainly composed of *Prunella* vulgaris, Kudzu root, *Plantago asiatica*, and *Lycium barbarum*. A total of 52 APIs were searched from the databases. The API-target network was constructed using Cytoscape3.8.0 (Figure 1(a)). Que, beta-sitosterol, and Kaempferol were the most connected targets in the network. After eliminating the duplicates, 2081 POAG-associated targets were identified in 5 databases (Figure 1(b)). From the comparative analysis between the POAG and QGLSF targets, 100 were obtained as QGLSF targets for the treatment of POAG (Figure 1(c)).

### 3.2. API-Target-POAG Network

The API-target-POAG network was constructed using Cytoscape3.8.0 (Figure 2). Analysis of the network revealed that 52 compounds and 100 targets played an important role in QGLSF's treatment of POAG. *Plantago asiatica* contained the most compounds in the network (Table 2). Among them, Que (*Prunella* vulgaris, *Plantago asiatica*, and *Lycium barbarum*) had the most intersections.

### 3.3. Hub Genes in PPI Networks

The PPI network was generated using STRING, showing a total of 308 nodes (Figure 3). Hub genes were filtered by median values of Betweenness, Closeness, Degree, Eigenvector, LAC, and Network scores using the CytoNCA plugin. After two rounds of screening, 9 hub genes were obtained, including ESR1, MAPK14, MYC, MAPK1, AKT1, JUN, RELA, FOS, and TP53.

### 3.4. KEGG and GO Enrichment Analyses

In the GO enrichment analysis, 2276 terms were obtained. As shown in Figure 4(a), the most involved biological processes mainly included the response to lipopolysaccharide, the response to molecules of bacterial origin, and the cellular response to chemical stress. The most involved cellular compositions included membrane rafts, membrane microdomains, and membrane domains. The most involved molecular functions included DNA-binding transcription factor binding, heme binding, and RNA polymerase II specific DNA-binding transcription factor binding.

KEGG enrichment analysis revealed 155 enriched signaling pathways, mainly including AGE-RAGE signaling pathway, fluid shear stress and atherosclerosis and prostate cancer (Figure 4(b)). The most significantly enriched pathway was the AGE-RAGE signaling pathway, which involved 25 hub genes, AKT1, VEGFA, BCL2, BAX, MMP2, and MAPK1 (Figure 5(b)). Using Cytoscape, a combination network was constructed with the top five pathways and the core targets (Figure 5(a)).

### 3.5. Que Enhanced the Activity of RGC-5 Cells Induced by CoCl_2_

To investigate the effect of Que on the viability of RGC-5, RGC-5 cells were pretreated with different doses of Que (0, 5, 12.5, 25, 50 *μ*M) for 24 h. The results showed that Que at 5, 12.5, 25, and 50 *μ*M enhanced the activity of RGC-5 cells (*p* < 0.05). Que at 25 *μ*M showed the strongest effect (*p* < 0.01) (Figure 6(a)). When the Que concentration rose to 50 *μ*M, the cell viability began to decrease. Therefore, Que concentrations of 12.5 and 25 *μ*M were chosen for subsequent experiments.

To confirm whether Que alleviated CoCl_2_-induced RGC-5 cell damage, CCK-8, and Annexin V-FITC assays were used to assess cell viability and apoptosis after pretreatment with Que and CoCl_2_. The results showed that CoCl_2_ significantly decreased the viability and increased the apoptosis of RGCs. However, after treatment with Que, the cell viability increased, with a peak at a concentration of 25 *μ*M (*p* < 0.01) (Figures 6(b) and 6(c)). However, the cell viability increased after the Que concentration reached 25 *μ*M (*p* < 0.05).

### 3.6. Que Inhibited Protein Secretion of Hub Genes

To validate the results of network pharmacology, we examined the expression of the proteins most enriched in the AGE-RAGE signaling pathway and some hub genes by ELISA. The results showed that CoCl_2_ increased the secretion of AGEs, RAGE, JUN, AKT-1, and TP53 in the cell supernatant. However, the secretion of AGEs, RAGE, JUN, AKT-1, and TP53 in the cell supernatant decreased significantly after treatment with Que, especially at the concentration of 25 *μ*M (Figure 7).

### 3.7. Que Inhibited mRNA Expression of Hub Genes

To further validate whether Que acts through targets and AGE-RAGE signaling pathway acquired by the network pharmacology, total RNA was extracted and mRNA expression of core genes was measured by RT-PCR. Since AGEs are a general term for a variety of proteins, their mRNA contents were measured in this study. The results showed that the mRNA expression of RAGE, AKT-1, JUN, and TP53 increased significantly after CoCl_2_ treatment, and the mRNA expression of RAGE, AKT1, JUN, and TP53 decreased significantly after Que treatment, especially at the concentration of 25 *μ*M (Figure 8).

## 4. Discussion

In this study, we validated the therapeutic mechanisms of QGLSF for POAG by means of network pharmacology and *in vitro* experiments. The network pharmacology analysis showed that the main API in QGLSF was Que. Que is a common flavonoid found in a variety of vegetables and fruits [17]. Owing to its strong antioxidative, anti-inflammatory, immunomodulatory, vascular-protective, and other biological activities, Que has been widely studied in the field of ophthalmology [18–20]. Que can penetrate the blood-brain barrier to exert its effects of antioxidation and neuroprotection [21, 22]. It has been found that Que can enhance the mitochondrial function of RGCs and inhibit mitochondria-induced apoptosis in vivo in a rat model of chronic ocular hypertension, thereby promoting the survival of RGCs [23]. In our study, Que significantly increased the viability and inhibited the apoptosis of RGC-5 cells treated with CoCl_2_. However, this efficacy should be warranted in clinical trials.

Through the PPI network, we obtained 9 hub genes targeted by QGLSF. These targets were mainly associated with inflammation and apoptosis. In the pathogenesis of POAG, RGC apoptosis can be caused by persistent high intraocular pressure [24]. The proapoptotic transcription factor JUN has been demonstrated to induce POAG-related neurodegeneration [25, 26]. JUN is a typical target of the JNK signaling pathway. Through this pathway, JNK phosphorylates and activates its canonical target, JUN, which in turn acts as a proapoptotic transcription factor by promoting the transcription of prodeath genes [27, 28]. In addition, JUN also acts on downstream EDN receptors to enhance ER stress response and mediate RGC death. Therefore, JUN may mediate RGC death as a response to EDN [29].

Protein kinase (AKT) is a human serine-threonine kinase and an AGC protein kinase with three highly homologous isoforms (AKT1, AKT2, and AKT3). AKT1 is expressed in a wide range of tissues [30, 31]. AKT1 is a key component of the phosphoinositide 3 kinase (PI3K)/AKT1 signaling cascade that can regulate cell growth and survival [32]. AKT mediates cell apoptosis via BCl2 and MDM2 pathways [33]. Recent studies have found that with primary cilia acting as sensors, AKT-1 interacts with SMAD2/3 to regulate the autophagy induced by mechanical stretch in trabecular meshwork cells [34]. Besides, the CD9/ITGA4/PI3K-Akt axis can mediate glaucomatous trabecular cell apoptosis through comprehensive transcriptional and proteomic analysis [35].

Tp53 is an inducible apoptotic nuclear transcription factor capable of inducing neuronal death and has demonstrated its implication in a variety of neurodegenerative diseases [36]. Studies have shown that the apoptosis-stimulating protein ASPP1/2 is abundantly expressed and promotes the expression of P53 in injured frontal RGC cells, which in turn induces apoptosis [37]. In the present study, we found that the expression levels of AKT-1, TP53, and JUN were all significantly increased in CoCl_2_-induced RGC-5 cells, but decreased after Que treatment. We speculate that Que may reduce the apoptosis of RGC-5 cells by inhibiting the expression of AKT-1, TP53, and JUN.

As shown in GO enrichment analysis, the response to lipopolysaccharide was the most significantly enriched. Lipopolysaccharide, as a potent endotoxin, can arouse systemic inflammation in many neurodegenerative diseases [38, 39]. The mechanism may involve the activation of the TLR-4 signaling pathways that increase the level of proinflammatory cytokines [40]. Excess lipopolysaccharide is deleterious to RGCs by inducing microglial activation, thus facilitating the progression of glaucoma [41]. Besides, stimulating microglia with lipopolysaccharide exacerbates optic nerve damage in rats with experimental glaucoma [42].

KEGG pathway enrichment analysis suggested that the hub genes were mostly involved in the AGE-RAGE signaling pathway. POAG is a multifactorial disease in which oxidative stress may play a major pathophysiological role. Meanwhile, oxidative stress is regulated by the AGE/RAGE signaling pathway [43, 44]. Studies have shown that AGEs can promote oxidative stress and mitochondrial dysfunction in ARPE-19 cells by interacting with RAGE, which in turn leads to apoptosis [45]. Moreover, the accumulation of AGEs and the activation of RAGEs sustain oxidative stress in vascular tissues [46]. The oxidative stress due to hyperglycemia promotes the formation of AGEs and the expression of RAGEs [47]. In addition, AGEs and RAGEs can activate PI3K/AKT signaling through HPA proteins [48, 49].

Through *in vitro* studies, we found that Que could reduce the levels of AGEs and RAGEs secreted by RGC-5 cells induced by CoCl_2_. It was found by RT-PCR that Que could similarly reduce the mRNA level of RAGEs induced by CoCl_2_ in RGC-5 cells, suggesting that Que may ameliorate CoCl_2_-induced RGC-5 cell damage through the AGE-RAGE signaling pathway.

There are some limitations in this study. First, we used the RGC-5 cell line to investigate the functional mechanism of glaucoma. Although commonly used in glaucoma-related research, this cell line may still lead to inaccurate results of experimental studies because of the possibility of contamination of the mouse photoreceptor cell line. Besides, we did not perform validation of APIs obtained in network pharmacology. Future validation of APIs by LC-MS/MS is still needed.

## 5. Conclusion

In this study, our network pharmacology analysis showed that Que may be the main API in QGLSF in treating POAG. *In vitro* experiments revealed that Que can significantly relieve CoCl_2_-induced RGC-5 cell injury. This mechanism may be that Que inhibits the expression of apoptosis-related genes (JUN, TP53, AKT1) through the AGE-RAGE signaling pathway. This study provides theoretical evidence for the efficacy of QGLSF in the treatment of POAG. However, clinical studies should be carried out to determine its dose and validate its efficacy in real-time settings.

## Figures and Tables

**Figure 1:** Screening of POAG and QGLSF-related targets and APIs. (a) API-target network. Red icons are targets and yellow icons are APIs. (b) Intersections in the venny diagram of POAG-related targets from Genecards, OMIM, PharmGKB, TTD, and Drugbank databases. (c) Intersections in the venny diagram of QGLSF and POAG targets.

**Figure 2:** The API-target-POAG network. Rectangles represent targets and circles represent active ingredients. Different colors in the circle represent different herbs (red represents *Plantago asiatica*, purple represents Kudzuvine root, orange represents *Lycium barbarum*, and green represents *Prunella* vulgaris).

**Figure 3:** PPI networks. (a) Initial PPI network; (b) secondary PPI network; (c) PPI network after final screening.

**Figure 4:** GO and KEGG enrichment analysis (a) GO enrichment analysis (b) KEGG enrichment analysis.

**Figure 5:** API-target-pathway network (a) API-target-pathway network. Yellow indicates target, green indicates API, and blue indicates pathway. (b) AGE-RAGE signaling pathways.

**Figure 6:** Cell viability and apoptosis assay. (a) Effect of different concentrations of que on RGC-5 cell viability. (b) Effect of que on CoCl_2_-inhibited RGC-5 cell viability. (c) Effect of que on CoCl_2_-induced apoptosis in RGC-5 cells. Values are represented as mean ± S.D. ^#^*p* < 0.05 versus control group. ^*∗*^*p* < 0.05 versus CoCl_2_ group. ^*∗∗*^*p* < 0.01 versus CoCl_2_ group.

**Figure 7:** Que regulated the expression of hub genes. (a) Expression of RAG in the cell supernatant. (b) Expression of AGEs in the cell supernatant. (c) Expression of AKT-1 in the cell supernatant. (d) Expression of JUN in the cell supernatant. (e) Expression of TP53 in the cell supernatant. Values are represented as mean ± S.D. ^#^*p* < 0.05 versus control group. ^*∗*^*p* < 0.05 versus CoCl_2_ group. ^*∗∗*^*p* < 0.01 versus CoCl_2_ group. ^*∗∗∗*^*p* < 0.001 versus CoCl_2_ group.

**Figure 8:** Que regulated the mRNA expression of core targets. (a) mRNA expression of RAG. (b) mRNA expression of TP53. (c) mRNA expression of JUN. (d) mRNA expression of AKT-1. Values are represented as mean ± S.D. ^#^*p* < 0.05 versus control group. ^*∗*^*p* < 0.05 versus CoCl_2_ group. ^*∗∗*^*p* < 0.01 versus CoCl_2_ group.

**Table 1:** RT-PCR primer sequences and product lengths.

Gene	Product length	Forward primer (5′ ⟶ 3′)	Reverser primer (5′ ⟶ 3′)
Gapdh	74	GCATCTTCTTGTGCAGTGCC	TACGGCCAAATCCGTTCACA
JUN	130	TGGGCACATCACCACTACAC	GGGCAGCGTATTCTGGCTAT
TP53	75	CCCCTGAAGACTGGATAACTGT	TCTCCTGACTCAGAGGGAGC
AKT1	101	GAACGACGTAGCCATTGTGA	AGGTGCCATCATTCTTGAGG
RAGE	140	ACAGAAACCGGTGATGAAGGA	TGTCGTTTTCGCCACAGGAT

**Table 2:** List of the top 10 genes and APIs.

Number	Gene name	Degree	MOL ID	Compound name	Degree
No. 1	PGR	31	MOL000098	Quercetin	84
No. 2	PTGS2	21	MOL000006	Luteolin	35
No. 3	PTGS1	17	MOL000422	Kaempferol	31
No. 4	NR3C2	16	MOL005406	Atropine	25
No. 5	NOS2	10	MOL000392	Formononetin	20
No. 6	AR	10	MOL009637	4-((Z,1R)-3-(4-Methoxyphenyl)-1-vinylprop-2-enyl) phenol	19
No. 7	ADRB2	8	MOL000358	Beta-sitosterol	18
No. 8	CHRM1	8	MOL000449	Stigmasterol	16
No. 9	DPP4	8	MOL008400	Glycitein	13
No. 10	PPARG	8	MOL002959	3′-Methoxydaidzein	11

## Data Availability

The data related to this research can be obtained from the corresponding author upon reasonable request.
